The article "Design of a tomato classifier based on machine vision" was retracted in 2025. Reason: compromised peer review.

# Design of a tomato classifier based on machine vision

**DOI:** 10.1371/journal.pone.0219803

**Published:** 2019-07-18

**Authors:** Li Liu, Zhengkun Li, Yufei Lan, Yinggang Shi, Yongjie Cui

**Affiliations:** College of Mechanical and Electronic Engineering, Northwest A&F University, Yangling, China; University College London, UNITED KINGDOM

## Abstract

This paper attempts to design an automated, efficient and intelligent tomato grading method that facilitates the graded selling of the fruit. Based on machine vision, the color images of tomatoes with different morphologies were studied, and the color, shape and size were selected as the key features. On this basis, an automated grading classifier was created based on the surface features of tomatoes, and a grading platform was set up to verify the effect of the classifier. Specifically, the Hue value distributions of tomatoes with different maturities were investigated, and the Hue value ranges were determined for mature, semi-mature and immature tomatoes, producing the color classifier. Next, the first-order Fourier descriptor (*1D- FD*) was adopted to describe the radius sequence of tomato contour, and an equation was established to compute the irregularity of tomato contour, creating the shape classifier. After that, a linear regression equation was constructed to reflect the relationship between the transverse diameters of actual tomatoes and tomato images, and a classifier between large, medium and small tomatoes was produced based on the transverse diameter. Finally, a comprehensive tomato classifier was built based on the color, shape and size diameters. The experimental results show that the mean grading accuracy of the proposed method was 90.7%. This means our method can achieve automated real-time grading of tomatoes.

## Introduction

Grading is a key measure to commercialize agricultural products, and thus improve the economic efficiency of agriculture [1]. The annual yield of tomatoes in China reaches 34 million tons [2], calling for the design of an automated tomato grading system that reduces intense manual labor and makes grading repeatable and accurate.

The automated tomato grading has been explored by various experts and scholars, using important indices like color, texture, size, shape and surface texture [3]. Many of them developed automated tomato grading algorithms based on computer vision [4]. For example, Pavithra V. et al. extracted the texture, color and shape features of tomato surface, and then realized the quality grading of mature tomatoes using the support vector machine (SVM) classifier based on K-nearest neighbors’ algorithm [5]. Peng Wang et al. recognized the color features of concentric circles with equal area on tomato surface, and created a maturity grading model based on these features and the backpropagation neural network (BPNN) [6]. Du Y. et al. put forward an edge detection algorithm based on fractional differential and Sobel operator, and proved its effect on the defect detection of cherry tomatoes through comparative analysis [7]. The methods of Pavithra V, Peng Wang and Du Y were useful for tomato detection with high accuracy, but the processing time is far away from meet sub-second analysis criteria. Arjenaki et al. took the eccentricity, mean color component and 2D pixel size of tomato images as the bases, and developed a machine vision-based tomato grading system capable of grading tomatoes by shape, maturity and size [8]. Arjenaki’ system achieves real-time classification, but a single camera obtains less surface features lead to unstable accuracy. Selman U. et al. took images of tomatoes from five angles using a high-definition digital camera, and estimated the fruit volume based on the horizontal and vertical distances of the tomato images [9]. Selman U’s work provides an approach to build 3D model of tomato, but that’s complex for automated grading. Overall, the above research is not effective in practice. So, the objective of our research is to develop a simple, real-time and efficient automated grading system for tomato based on machine vision.

The article "Design of a tomato classifier based on machine vision" was retracted in 2025. Reason: compromised peer review.

Before making a buying decision, the consumer often evaluates the tomatoes by such surface features as color, size and shape. In view of this, the author designed a grading algorithm based on the color, size and shape features of tomatoes according to the Chinese agricultural standard Grades and Specifications of Tomatoes (NY/T 940–2006). Next, the proposed algorithm was applied to a grading system based on machine vision, and verified by an experiment. The results show that the proposed method is feasible. The research findings shed new light on the automated grading of tomatoes.

## Materials and methods

### Selection of Tomato Grading Features

In the NY/T 940–2006 [10], the size of tomatoes is classified by the transverse diameter of the fruit, i.e. the diameter of the largest cross-section. If the transverse diameter is greater than 7 cm, the tomato is allocated to the large (L) category; if it falls between 5 cm and 7 cm, the tomato belongs to the medium (M) category; if it is smaller than 5 cm, the tomato is added to the small (S) category.

The NY/T 940–2006 divides tomatoes into special, first second and unqualified grades based on the variety feature, shape, color, maturity, hardness, disease and pest injury, as well as other injuries. The specific criteria are detailed below:

Special grade: Consistent appearance, round and rib-free (except for ribbed varieties) fruit, moderate and consistent maturity, uniform color, smooth surface, small cavity, good elasticity, no damage, no crack, no scar;

First grade: Basically consistent appearance, basically round and slightly deformed fruit, maturity or slight under-ripeness, basically consistent maturity, relatively uniform color, slight defects on the surface, small cavity, good hardness and elasticity, no damage, no crack, no scar;

Second grade: Basically consistent appearance, basically round and slightly deformed fruit, slight under- or over-ripeness, relatively uniform color, medium cavity, relatively high hardness, poor elasticity, slight damages, no crack, slight scars on the peel, unaffected commercial properties;

Unqualified grade: inconsistent appearance, deformed fruit, under- or over-ripeness, uneven color, severe defects on the surface, large cavity, poor hardness and elasticity, severe damage, severe crack, severe scar.

The article "Design of a tomato classifier based on machine vision" was retracted in 2025. Reason: compromised peer review.

It can be seen that the tomatoes are mainly graded by sensory factors. Among the above grading features, there is a certain correlation between maturity, color, hardness and elasticity of the tomato. However, these features cannot be clearly differentiated by visual classification alone. For simplicity, these feature indices are replaced with the color feature of tomato images in our research. Since the surface defects of tomatoes are too complex to be detected accurately, this paper takes color, shape and size features as the bases for tomato grading.

### Extraction of Tomato Grading Features

#### Image processing

The color, size and shape are surface features of tomatoes. To extract and analyze these feature data, the tomato image was taken by an MD-GED130C-T camera and subjected to processing. The flow of image acquisition and processing is illustrated in Fig 1. First, the original image of the target tomato was taken directly by the camera; Next, the image went through enhancement, filtering and morphological processing, aiming to eliminate the background interference and ensure the segmentation accuracy; After that, the fruit was separated from the background based on the surface color.

**Fig 1:** The flow chart of image acquisition and processing.

The original image and the images generated in each step of processing are presented in Fig 2. As shown in Fig 2(a), the tomato image taken by the camera has a high gray value due to the high intensity of the ring light source. Thus, the color of the original image was corrected by the standard color plate, and the image contrast was enhanced through Gamma transform [11], yielding the image in Fig 2(b). Next, the image was filtered by the high-speed median filter based on neighborhood processor [12], with the aim to suppress noise and preserve key information like contour and edges. The resulting image is shown in Fig 2(c). After that, the RGB (red, green, blue) image was converted into the HSV (hue, saturation, value) image (Fig 2(d)). Subsequently, the fruit area was differentiated from the white background by Otsu’s segmentation method [13]. The resulting image in Fig 2(e) was subjected to the open and closed operations in morphological filtering [14] to eliminate tiny discrete closed regions and boundary interference in the white background. The filtered image is displayed in Fig 2(f). Under the reflection of tomato pedicle and surface, the interior of the highlighted area of the fruit may be mistaken for the black background. To solve the problem, multiple contours were identified by looking for discontinuities of pixel gray value on the boundary between the highlighted area and the black area, and the maximum contour was extracted to be the tomato contour (Fig 2(g)). Finally, the tomato fruit was separated from the image by selecting the pixels inside the contour (Fig 2(h)).

The article "Design of a tomato classifier based on machine vision" was retracted in 2025. Reason: compromised peer review.

**Fig 2:** The original image and the images generated in each step of processing. (a) Original Image; b) Gamma Transform; c) Median Filtering; d) HSV Transform; e) OTSU Segmentation; f) Morphological Treatment; g) Find Contours; h) Processing Result).

#### Maturity judgement

The HSV color model describes the color with three parameters: hue (H), saturation (S) and value (V). These parameters are visually independent of each other, and compatible with the visual features of our eyes in spatial distance. In a stable environment, the S and V are constant, and the fruit color can be characterized by the H [15]. Hence, H was extracted for the analysis of tomato color.

The H in the HSV image can be depicted by the Hue value, which ranges from 0° to 180° in the Open Source Computer Vision Library (OpenCV). Here, the surface colors of mature, semi-mature and immature tomatoes are statistically analyzed by Hue histogram. The results in Fig 3 show that the Hue values of mature tomatoes concentrated in 0°~8° or 170°~180°, those of semi-mature tomatoes in at 8°~20°, and those of immature tomatoes at 40°~67°. There are marked differences in Hue value between tomatoes with different maturities. In view of this, a tomato maturity classifier was designed to determine the threshold range of Hue value of tomato surface color, thus judging the fruit maturity:

$$H\text{ue}=\{\begin{array}{l} 0\sim 8\;\text{or}\;170\sim 180,\;mature\;tomatoes\\ 8\sim 20,\;semi-mature\;tomatoes\\ 40\sim 67,\;raw\;tomatoes \end{array}$$ (1)

**Fig 3:** Hue histograms of tomatoes with different maturities.

The article "Design of a tomato classifier based on machine vision" was retracted in 2025. Reason: compromised peer review.

Next, 120 tomatoes, including 83 mature ones, 29 semi-mature ones and 8 immature ones, were selected and graded three times by the said tomato maturity classifier. The grading results are listed in Table 1 below. Obviously, the classifier achieved a mean accuracy of 92.8%, indicating that it can be used for the maturity grading of tomatoes.

**Table 1:** Grading results of tomato maturity classifier.

Machine detection				Errors	Accuracy
Times	Mature	Semi-mature	Immature		
1	80	23	9	8	93.3%
2	78	24	9	9	92.5%
3	77	25	9	9	92.5%

#### Shape judgement

The Fourier descriptor (FD) is the most commonly used descriptor in the existing boundary shape representation methods [16]. In this paper, the contour-based the first-order Fourier descriptor (1-D FD) is employed to process the closed contour in the original image, and the resulting Fourier coefficient is taken as a vector to characterize the target shape. Then, the 2D target shape was transformed into a 1D function, which in turn quantifies the shape of the target tomato.

The Hu moment, as a geometric moment, can describe the features of an image. Let f(x, y) be the function of the target image. Then, the p+q-order moment of a W×H discrete image can be expressed as:

$$m_{pq}=\sum_{\text{y}=1}^{\text{H}}\sum_{\text{x}=1}^{\text{W}}x^{p}y^{q}f(x,y)$$ (2)

The zero-order moment of the binary image m00 represents the connected domain area of the contour. Using the zero- and first-order moments, the coordinates (xc, yc) of the center point of the contour in the image can be calculated as:

$$\begin{array}{l} x_{c}=m_{10}/m_{00}\\ y_{c}=m_{01}/m_{00} \end{array}$$ (3)

The radius sequence from (xc, yc) to the boundary points of the contour (xk, yk) can be computed as:

$$r_{k}={\left[{\left(x_{k}-x_{c}\right)}^{2}-{\left(y_{k}-y_{c}\right)}^{2}\right]}^{\frac{1}{2}}$$ (4)

For the fruit contour in Fig 2(g), the Hu moment of the image was computed by Eq (2), the coordinates of the geometric center [17] of the tomato contour was obtained by Eq (3), and the radius sequence from the center point to the boundary points of the contour was derived from Eq (4). After that, the radius sequence went through discrete Fourier transform below:

$$F(\omega )=\frac{1}{n}\sum_{k=0}^{n-1}r_{k}\text{exp}[-j\frac{2\pi k\omega }{n}]=\frac{1}{n}\sum_{k=0}^{n-1}r_{k}[\text{cos}(-\frac{2\pi k\omega }{n})+j\text{sin}(-\frac{2\pi k\omega }{n})]$$ (5)

where w is frequency; n is the number of sequence points; rk is the radius sequence. The Fourier mode |*F*(*ω*)| is called the Fourier coefficient. The value of |*F*(*ω*)| continues to decrease with the growth in frequency w. The Fourier coefficient becomes so small as negligible after w surpassed 10.

The article "Design of a tomato classifier based on machine vision" was retracted in 2025. Reason: compromised peer review.

Next, the ten terms with the largest |*F*(*ω*)| values were subjected to the inverse Fourier transform. The resulting boundary images are basically the same as the original image. Among the shapes implied by the Fourier coefficient, F(0), F(1), F(2), F(3) and F(4) respectively refer to the mean radius, curvature, elongation, triangle and rectangle. Thus, F(w) can be understood as the variation in the radius sequence after changing w times. The greater the F(w) value, the more irregular the shape of the target. Let |*F*(*ω*)| be the L components with the largest Fourier coefficients out of the first k components. Then, the boundary irregularity s can be judged by:

$$s=\sum_{i=0}^{L}\left|F_{i}(\omega )\right|\omega^{m}(m\in \{1,2,3\})$$ (6)

Here, the radius sequence undergoes the Fourier transform by Eq (5), and the mathematical expression of tomato shape irregularity is constructed by Eq (6). With this expression, the different contour shapes were transformed into varied irregularities, laying a solid basis for irregularity testing of tomatoes.

The boundary changes are reflected in F(w). Thus, the shape is more irregular with the increase of the s value. The tomatoes of different shapes can be differentiated more clearly by adjusting the value of the description coefficient m. Fig 4 shows the typical contour images of tomatoes, where contours (a) and (b) were extracted from the images on round tomatoes, contours (c) and (d) from the images on generally shaped tomatoes, and contours (e) and (f) from the images on poorly shaped tomatoes.

**Fig 4:** The typical contour images of tomatoes.

The center point of each typical contour in Fig 4 was computed by the Hu moment. Then, the radius sequence of each contour was calculated, and substituted into Eqs (4) and (5). The shape irregularities s was obtained with the description coefficient m being 1, 2 or 3. The results in Table 2 show that the boundary irregularity s increased with the shape irregularity of tomatoes; the larger the m value, the more enhanced the high-frequency components. When m = 3, the round, generally-shaped and poorly-shaped fruits differed greatly in irregularity.

**Table 2:** The shape irregularities of different shaped tomatoes.

Contours	a	b	c	d	e	f
**m = 1**	11.57	16.32	24.37	26.62	32.12	43.63
**m = 2**	41.96	63.36	100.36	116.35	182.33	287.52
**m = 3**	206.21	357.44	670.33	806.63	1386.55	2304.59

In order to verify the feasibility of using the irregularity function to classify shapes, 15 round tomatoes, 15 generally-shaped tomatoes and 15 poorly-shaped tomatoes were selected, and the contour of each tomato was extracted. Taking m = 3, the irregularities s of these tomatoes was calculated by Eq (6). The tomatoes with *s* ≤ 500 were defined as round ones, those with 500 ≤ *s* ≤ 1000 as generally-shaped ones and those with *s* ≥ 1000 as poorly-shaped ones. The results in Table 3 show that the shape classifier achieved the mean accuracy of 91.1%.

The article "Design of a tomato classifier based on machine vision" was retracted in 2025. Reason: compromised peer review.

**Table 3:** Grading results of tomato shape classifier.

Machine Detection				Errors	Accuracy
Times	Round Shape	General Shape	Poor Shape		
1	13	2	0	2	86.6%
2	1	14	0	1	93.3%
3	0	1	14	1	93.3%

#### Size judgement

The tomato size depends on the maximum transverse diameter. Based on the principle of monocular image sequence, when both the camera parameters as well as the distance between the tomato and camera are fixed, image size is positively linear to actual size. The size threshold is clearly proposed for grading in the NY/T 940–2006 and a model was put forward to describe the shifting relationship between the reality and images.

Firstly, the tomato sample images were collected, the transverse diameters of the images and actual tomatoes were measured, and then the mapping between the image size and the actual size was established. After that, the maximum transverse diameters were measured in the images of the target tomatoes. Based on the mapping and maximum values, the grading system could divide the tomatoes into large, medium and small categories.

To verify the feasibility of above method, we selected a CCD camera with a focal length of 3.6mm and a maximum resolution of 1920*1080. The vertical distance between the tomato and the camera is 230 mm. The author took 112 tomato samples and measured their maximum transverse diameters Wr. Then, the diameter of the minimum circumscribed circle (MCC) of each image contour was obtained by Graham scan, one of finding the minimum perimeter convex hull method. Taking the MCC diameter as the maximum transverse diameter Wp of the tomato image, a linear regression model was constructed between Wr and Wp (Fig 5):

$$W_{r}=0.264W_{p}+20.597$$ (7)

where the correlation coefficient *R*^*2*^ = 0.903; the p-value is smaller than 0.001. Thus, the said model is sufficiently accurate to meet experimental requirements.

**Fig 5:** Linear regression model of tomato size.

According to the NY/T 940–2006, the transverse diameter that differentiates between large and medium tomatoes and that between medium and small ones are respectively 7 cm and 5 cm. Substituting the data into the regression Eq (7), the maximum transverse diameter Wp that differentiates between large and medium tomatoes and that between medium and small ones can be determined as 111 and 187 pixels, respectively. On this basis, the author set up a classifier that divides tomato fruits into large, medium and small categories.

The article "Design of a tomato classifier based on machine vision" was retracted in 2025. Reason: compromised peer review.

To verify the performance of our size classifier, 100 large tomatoes, 100 medium tomatoes and 100 small tomatoes were selected. An image was taken for each tomato and prepressed. Then, the transverse diameter Wp of each image was computed and substituted into the proposed size classifier. The grading results in Table 4 show that the mean grading accuracy was 92.6%, a proof for the feasibility of the size classifier.

**Table 4:** Grading results of tomato size classifier.

Machine Detection				Errors	Accuracy
Times	Large	Medium	Small		
1	96	4	0	4	96.0%
2	8	87	5	13	87.0%
3	0	5	95	5	95.0%

#### Design of comprehensive classifier

In the NY/T 940–2006, tomatoes are classified into four grades, namely, the special grade, the first grade, the second grade and the unqualified grade. Each grade is further split into subgrade of large, medium and small grade based on the tomato size. Following this train of thought, a comprehensive classifier was designed to determine the tomato grade through overall consideration of the color, shape and size features. The flow of the comprehensive analysis is illustrated in Fig 6. First, the color and shape features were extracted from tomato images, to judge if the maturity and shape are as required. Among the tomatoes meeting the maturity and shape requirements, the mature and round ones were classified to the special grade, the mature and general-shaped ones to the first grade, and the rest to the second grade. Finally, the tomato size features were extracted to divide the tomatoes into large, medium and small classes.

**Fig 6:** The flow of the comprehensive analysis.

The grading criteria are as follows: the tomatoes with Hue values in 0°~8° or 170°~180° were considered mature, those with Hue values in 8°~20° were considered semi-mature, and those with Hue values in 40°~67° were considered immature; a large tomato must have more than 187 pixels on the maximum transverse diameter in its image, a medium tomato must have 111~187 pixels on the maximum transverse diameter in its image, and a small tomato must have fewer than 111 pixels on the maximum transverse diameter in its image; when the description coefficient m = 3, the tomatoes were deemed as round if the contour irregularity s is smaller than 500, generally-shaped if s is between 500 and 1,000, and poorly-shaped if s is greater than 1,000.

#### Experimental platform

To test the accuracy of the comprehensive classifier, an automated tomato grading system was built as Fig 7. When a tomato passes through the conveying mechanism 1, the photoelectric sensor in the visual inspection box 2 will detect it and make a change to high level, which will be received by microcomputer 5; then, the camera is triggered to take an image of the tomato. Next, the feature information of the image is extracted, and the tomato is graded by the comprehensive classifier. The grading result will be transmitted to the PLC controller 4, which controls the grading execution mechanism 3 to complete the grading of tomatoes. Meanwhile, the grading results will be displayed on the computer screen. The microcomputer 5 belongs to the GK1037 series, running on Intel Core i5-3317U CPU and Ubuntu 16.04 LTS.

The article "Design of a tomato classifier based on machine vision" was retracted in 2025. Reason: compromised peer review.

**Fig 7:** Automated tomato grading system. (1. Conveying mechanism; 2. Visual inspection box; 3. Grading execution mechanism; 4. PLC controller; 5. Microcomputer).

The structure of the visual inspection box is described in Fig 8. Specifically, the ring light source 2 provides a lighting environment. When the photoelectric sensor 1 detects that a fruit passes through the conveyor belt, three cameras will take images of the tomato to obtain image information of the tomato surface.

**Fig 8:** Structure of the visual inspection box. (1. Photoelectric sensor; 2. Ring light source; 3. Camera).

The upper computer software was compiled on VC++ in Linux, which triggers the camera to take images of the tomatoes, and processes the image information with OpenCV. The operation interface of the software is presented as Fig 9.

**Fig 9:** The operation interface of computer software.

#### Experimental results

A total of 100 Jinpeng No. 11 tomatoes, which are produced in northwestern China’s Shaanxi Province, were selected randomly for our experiment. All tomatoes were transmitted with the pedicle pointing towards the conveying direction, making it easier for the camera to take images. Then, the proposed comprehensive classifier was adopted to grade these tomatoes in the grading system, and the grading results were displayed on computer software. After testing, the average processing time of each tomato was 0.0687s. The experiment was repeated three times and the grading results are recorded in Table 5. The experimental results show that the mean grading accuracy stood at 90.7%.

**Table 5:** The experimental results.

Grade	Size	Standards	Times of Machine detection		
			1	2	3
**Super-grade**	**Large**	11	13	12	12
	**Medium**	7	6	8	10
	**Small**	5	4	5	4
**First-grade**	**Large**	16	14	13	14
	**Medium**	21	19	16	18
	**Small**	7	9	8	8
**Second-grade**	**Large**	6	7	9	8
	**Medium**	7	8	9	6
	**Small**	7	9	7	8
**Unqualified**		13	11	13	12
**Error**			9	10	8
**Accuracy**			91.0%	89.0%	92.0%

The article "Design of a tomato classifier based on machine vision" was retracted in 2025. Reason: compromised peer review.

## Conclusions

Taking maturity, size and shape as the grading bases, this paper probes into the computer vision-based tomato grading according to the NY/T 940–2006, designs a grading algorithm considering the surface features, and builds a grading experimental platform to verify the algorithm.

Specifically, the color features of tomatoes with different maturities were obtained using the histograms of color HSV model, creating a maturity classifier; the irregularity function s of tomatoes with different sizes was established based on the first-order FD shape description method, producing the shape classifier; the regression equation between the transverse diameters of actual tomatoes and tomato images was set up, leading to the size classifier. The three classifiers were combined into a comprehensive classifier for tomato grading. Then, the experimental platform was created to test the comprehensive classifier. The feasibility of the proposed method was proved by the mean grading accuracy of 90.7%. This means our method can achieve automated real-time grading of tomatoes.

## Discussion

A specific variety of tomatoes named Jinpeng No. 11, which was widely planted in Shaanxi, China, was selected to inspect grading models in all the experiments. We researched a practical method for tomato grading according the standard of NY/T 940–2006, but those specific grading parameters should be adjusted depending on the operation especially in variety. This paper provides practical methodology and reference for automated real-time grading of other fruits.

However, there is still ample room for improving the grading accuracy of the proposed method. After all, the grading accuracies of shape and size are constrained by the changing relative positions between the tomatoes on the conveyor belt and the camera, and the image color may be distorted by the effect of light intensity on camera initialization. The proposed method is now only applicable to detect and grade the quality of tomato fruits one by one on the conveyor belt.

In addition, defect, PH, acid and sugar content detection are considered as the important factors in fruit grading according previous research, which are mostly based on spectral analysis and can’t meet the sub-second analysis criteria in practice. The further research will try to overcome this limitation.

## Supporting information

S1 File Additional instructions for verification experiments. (DOCX)

S2 File Original data. (RAR)

S3 File Data availability. (TXT)

S4 File Funding information. (TXT)
